The article "Ameliorative Impact of Liraglutide on Chronic Intermittent Hypoxia-Induced Atrial Remodeling" was retracted in 2023. Reasons: signs of a paper mill; suspected computer-generated content; unreliable results or conclusions; concerns about the data.

# Ameliorative Impact of Liraglutide on Chronic Intermittent Hypoxia-Induced Atrial Remodeling

**DOI:** 10.1155/2022/8181474

**Published:** 2022-04-13

**Authors:** Jun Wang, Yongzheng Liu, Changhui Ma, Yue Zhang, Meng Yuan, Guangping Li

**Affiliations:** Tianjin Key Laboratory of Ionic-Molecular Function of Cardiovascular Disease, Department of Cardiology, Tianjin Institute of Cardiology, The Second Hospital of Tianjin Medical University, Tianjin 300211, China

## Abstract

Atrial fibrillation (AF) is the most frequent form of clinical cardiac arrhythmias. Previous evidence proved that atrial anatomical remodeling (AAR) and atrial electrical remodeling (AER) are crucial for the progression and maintenance of AF. This study is aimed at investigating the impact of the glucagon-like peptide-1 (GLP-1) receptor agonist, Liraglutide (Lir), on atrial remodeling (AR) mouse model induced by chronic intermittent hypoxia (CIH). C57BL/6 mice were categorized randomly into the control, Lir, CIH, and CIH+Lir groups. CIH was performed in CIH and CIH+Lir groups for 12 weeks. Lir (0.3 mg/kg/day, s.c) was administered to the Lir and CIH+Lir groups for four weeks, beginning from the ninth week of CIH. Meanwhile, echocardiography and right atrial endocardial electrophysiology via jugular vein, as well as induction rate and duration of AF, were evaluated. Masson and Sirius red staining assays were utilized to assess the extent of fibrosis in the atrial tissue of the mice. Immunohistochemical staining, RT-qPCR, and Western blotting were performed to evaluate the marker levels of AAR and AER and the expression of genes and proteins of the miR-21/PTEN/PI3K/AKT signaling pathway, respectively. ELISA was also performed to evaluate the changes of serum inflammatory factor levels. The CIH group exhibited significant AR, increased atrial fibrosis, and a higher incidence rate of AF compared to the control group. Lir could significantly downregulate the protein expression level in the PI3K/p-AKT pathway and upregulated that of phosphatase and tensin homolog deleted on chromosome ten (PTEN). Moreover, Lir downregulated the expression of miR-21. However, the protein expressions of CACNA1C and KCNA5 in atrial tissue were not changed significantly. In addition, Lir significantly attenuated the levels of markers of inflammation (TNF-*α* and IL-6) in the serum. In the mouse model of CIH, Lir treatment could ameliorate AR by the miR-21/PTEN/PI3K/AKT signaling pathway and modulation of inflammatory responses.

## 1. Introduction

Atrial fibrillation (AF) is the most frequent form of clinical cardiac arrhythmia [1]. With an enhancive population of elderly and an enhanced proportion of comorbidities, the incidence of AF along with disabling thromboembolic disease is increasing [2, 3], thereby worsening the quality of life of patients. The healthcare expenditure has become exorbitant [4]. AF pathogenesis processes are complex and remain unclear. Nevertheless, the available evidence suggests that atrial anatomical remodeling (AAR) and atrial electrical remodeling (AER) are crucial for the progression and maintenance of AF [5, 6].

Obstructive sleep apnea (OSA) is recognized as an important risk factor for AF [7]. Iwasaki et al. [8] investigated the effect of acute OSA on susceptibility to AF in rats and showed that forced inspiration-induced acute left atrial dilation and diastolic dysfunction may underlie the mechanisms of AF progression. In addition, several clinical studies demonstrated that OSA is correlated with a greater risk of AF relapse following catheter ablation and cardioversion [9, 10]. A study demonstrated that [11] in canine model, chronic OSA caused chronic intermittent hypoxia and could shorten AERP, lead to altered expression of important channel proteins, and then caused AER. Moreover, CIH induced AAR by increased atrial apoptosis, fibrosis, and autonomic remodeling. AER and AAR are important substrates of atrial fibrillation. AR increases the susceptibility and recurrence rate of atrial fibrillation [5, 6]. In this study, a mouse model of the chronic intermittent hypoxia- (CIH-) induced AF was established. As a major pathophysiological disorder of OSA, CIH is closely associated with multisystem diseases, especially AF [12].

Glucagon-like peptide-1 (GLP-1), a glucagon-like peptide hormone, is secreted by the intestinal L cells. It inhibits glucagon secretion, reduces postprandial hyperglycemia, delays gastric emptying, and stimulates insulin secretion [13]. Liraglutide (Lir), a long-acting GLP-1 receptor agonist having 97% sequence identity to human GLP-1, has been widely applied in the therapy of type 2 diabetes [14]. In addition to glucose regulation, a recent study showed that GLP-1R agonists result in other biological effects, particularly protective effects against various cardiovascular diseases unrelated to glucose regulation, such as improvement in cardiac function, amelioration of cardiomyocyte injury, regulation of blood pressure, and protection of vascular endothelial cell function [15]. Gaspari et al. [16] showed that Lir can attenuate interstitial myocardial fibrosis in several pathological conditions. Nakamura et al. [17] reported that Lir could suppress electrophysiological changes, reduce the incidence rate of AF, and decrease conduction velocity in canine model of AF. Early administration of Lir in C57BL/6 mice following ischemia-reperfusion reduced ROS production in the heart, inhibited proinflammatory cytokine signaling pathways, and attenuated collagen deposition [18]. Although these studies suggested a role of Lir in cardiovascular diseases, its effects on CIH-induced AR have not yet been reported. Hence, we reasonably speculated that Lir may ameliorate CIH-induced AR by modulating the PI3K/AKT signaling pathway and attenuating inflammatory responses.

## 2. Materials and Methods

### 2.1. Protocols for Animal Experiments

The study design was approved by the Experimental Animal Administration Committee of Tianjin Medical University (approval number: TMUaMEC2016012). Our experiments complied with the ARRIVE guidelines. Male C57BL/6J mice (Hufukang Biotechnology Co. Ltd., Beijing, China), 8–10 weeks old, were procured. All mice were maintained in a controlled environment (20 ± 2°C; 12 h : 12 h light : dark cycle), provided water ad libitum, and fed on a standard chow diet. The male C57BL/6 mice were categorized randomly into four groups based on the treatment condition as follows: control, Lir, CIH, and CIH with Lir treatment (CIH+Lir) groups. CIH was induced using an automated system (GC-A01, Maworde Industry and Trade Co, Ltd., Heilongjiang, China) that controlled the ambient oxygen concentration [19]. This system cycled the oxygen concentration between 18% and 6% by alternatively filling with 100% nitrogen (the oxygen concentration reduces gradually to 6%) and then filling with oxygen (its concentration increases to 18% gradually). CIH was induced for 8 h/d for 12 weeks. Lir administration (0.3 mg/kg/day, s.c, Novo Nordisk A/S, Bagsvaerd, Denmark) in the Lir and CIH+Lir groups was initiated in the ninth week of CIH. The treatments were performed for four weeks.

### 2.2. Measurements of Blood Pressure and Echocardiography

After four weeks of Lir administration, the blood pressure (BP) of conscious animals was recorded using the tail-cuff plethysmography (BP-98A, Softron Corporation, Beijing, China). The measurements were recorded in preheated chambers at 36–37°C for 10–15 min following the training sessions.

Using the Vevo 2100 system with an MS400 linear array transducer (VisualSonics, ON, Canada), the procedure of transthoracic echocardiography was performed on all mice. Briefly, mice were anesthetized using 2% isoflurane and kept warm using a heating pad (37°C). A depilatory cream was used to remove the chest hair, and a layer of acoustic coupling gel was applied to the thoracic region. RVFWT was measured from the parasternal short-axis view at the midpapillary level of the left ventricle. The pulmonary blood outflow was recorded by pulse-wave Doppler echocardiogram at the level of the aortic valve in the short axis view to measure the values of PAT, PET, and mPAP. Next, the LAD, the left ventricular ejection fraction (LVEF), and LVEDD were measured as described previously [20].

### 2.3. Induction of AF and Mapping of Atrial Epicardial Activation

2.5% tribromoethanol (0.02 mL/g; Sigma-Aldrich, United Kingdom) was used to anesthetize the mice. The electrophysiological measures were recorded as described previously [21]. Briefly, a 1.1F octupole electrophysiology catheter (Millar Instruments, EPR-800, USA) was inserted through the right jugular vein and advanced into the right atrium. The catheter consisted of eight poles; seven poles of the electrodes recorded atrial electrocardiograms (ECGs), and one pole was for pacing. Standard surface ECG lead II and seven right atrial ECGs were recorded on the PowerLab data acquisition system (ADInstruments, Shanghai, Co). The atrial arrhythmia inducibility was evaluated by applying 20-second-burst pacing using the catheter electrodes; this was repeated five times in 60-second intervals. The duration of subsequent AFs after each burst pacing was recorded. AF was defined as the rapid, irregular atrial, and ventricular responses longer than 1000 ms.

After anesthetizing, endotracheal intubation and mechanical ventilation were performed under strictly aseptic operation conditions and the heart was fully exposed after thoracotomy. For recording conduction signals, during the spontaneous and normal beating of the heart, a 36-microelectrode (configuration of 6 × 6) was placed on the epicardial surface of the atrium. The filter amplifier amplified the activation waveform and transmitted it to the computer. The Electric Mapping Scope System (MappingLab, UK) was used to acquire and digitize the atrial epicardial activation maps. The point, wherein the negative slope of the activated waveform was the maximum, was the activation time. The EMapScope analysis software (version: 4.0) (MappingLab, UK) was used to determine the values of absolute inhomogeneity, inhomogeneity index, and epicardial conduction velocity of the atrium.

### 2.4. Histological Assay

Using 10% neutral-buffered formalin, the tissues were fixed for 72 h at room temperature and subsequently embedded by paraffin. 5 *μ*m thick heart tissue sections were stained. To evaluate the structural diversity in cardiac myocytes, hematoxylin-eosin (H&E) staining (Solarbio Life Sciences, Beijing) was performed. Collagen deposition was measured by Sirius red and Masson's trichrome staining assays following the kit protocol (Solarbio Life Sciences, Beijing). To evaluate the protein level expressions of PTEN, PI3K, AKT, and p-AKT in the atrial tissues, immunohistochemistry (IHC) assays were performed. Briefly, antigen retrieval is by boiling in sodium citrate buffer (pH 6.0) for 15 min. Block endogenous peroxidase by 3% hydrogen peroxide for 20 minutes. Block buffer (normal goat serum) at 37°C for 30 min, followed by incubation with primary antibodies PTEN (bs-0686R, Bioss Co. Ltd., Beijing, China), p-AKT (bs-0876R), PI3K (bs-10276R), and AKT (bs-0115R) at 4°C overnight, followed by a conjugated secondary for 20 minutes and DAB staining. The Olympus inverted microscope (IX53, Tokyo) was used to capture the images of the sections, and the stained images were digitized and analyzed using the ImageJ software (version: 1.53, Media Cybernetics, Rockville, MD, USA).

### 2.5. Western Blotting

Using RIPA lysis buffer with PhosSTOP (#04906845001, Roche, IN), the total proteins were extracted from the atrial tissue and quantified using the BCA Protein Assay Kit (Thermo Fisher Scientific, MA). Next, the samples (20 *μ*g protein) were separated on the SDS-PAGE gel, and these proteins were transferred onto a PVDF membrane. After blocking with TBST buffer with 5% bovine serum albumin, the PVDF membranes were incubated overnight at 4°C with the following primary antibodies: tubulin (1 : 2000, Abcam, USA), GAPDH (1 : 5000, Abcam), collagen I (1 : 500, Abcam), collagen III (1 : 1000, Bioss, China), ɑ-SMA (1 : 1000, Abcam), PTEN (1 : 1000, Abcam), p-AKT (1 : 1000, Cell Signaling Technology, USA), PI3K (1 : 1000, Cell Signaling Technology), AKT (1 : 1000, Cell Signaling Technology), CACNA1C (1 : 1000, Bioss, China), KCNA5 (1 : 1000, Bioss, China), and CX43 (1 : 1000, Bioss, China). These membranes were washed thrice with 1× TBST buffer followed by incubation with HRP-labeled secondary antibodies (goat anti-rabbit and anti-mouse) for 1 h at room temperature. ImageJ was used to digitize and measure the optical intensities of the protein bands relative to those of tubulin or GAPDH.

### 2.6. RT-qPCR

The Eastep Super Total RNA Extraction Kit (LS1040, Promega, WI) was used to extract the total RNA. Using the iScript cDNA Synthesis Kit (Bio-Rad, CA), cDNA was synthesized. The real-time fluorescent quantitative PCR was performed on the 7500 Real-Time PCR System (Life Technologies, USA). The 2^-*ΔΔ*Ct^ method was utilized to draw the comparisons among mRNA levels, following the cycle threshold (Ct) data collection. The primers used in this experiment are listed in Table 1.

### 2.7. ELISA

TNF-*α* and IL-6 levels were assessed using an ELISA kit (Mlbio, Shanghai) per the manufacturer's protocol.

### 2.8. Statistical Analysis

Data were presented as mean ± standard error of the mean (SEM). One-way ANOVA with Bonferroni multiple comparison post-hoc-tests was used to analyze the significant differences. The criterion for statistical significance was set at *P* < 0.05. All statistical analyses were performed using GraphPad Prism 7 v7.04 (GraphPad Software, Inc., California, USA).

## 3. Results

### 3.1. Effects of Liraglutide on Heart/Body Weight, Heart Rate, Blood Pressure, and Blood Glucose in CIH Mice

No statistical differences were observed in heart weight/body weight (HW/BW) and heart rate between the four groups. The SBP level was increased in the CIH group compared with the control group (*P* < 0.05). The body weight (BW), SBP, and DBP were decreased in the Lir group compared with the control group (*P* < 0.05). The BW, blood glucose, SBP, and DBP were decreased in the CIH+Lir group compared with the CIH group (*P* < 0.05). Particularly, CIH substantially increased SBP. The hypotensive effect of Lir was demonstrated by the reduction in SBP and DBP levels in all groups following Lir administration (Figures 1(a)–1(f)and Supplementary Table 1).

### 3.2. Echocardiography

There were increases in the mean pulmonary artery pressure (mPAP) and right ventricular free wall thickness (RVFWT), while pulmonary artery acceleration time (PAT) and PAT/pulmonary ejection time (PET) decreased significantly in the CIH group compared to the control group (*P* < 0.05). Following the Lir administration, these indices were ameliorated significant statistically. Moreover, there were no statistical differences among the four groups in left ventricular end-diastolic diameter (LVEDD), left ventricular ejection fraction (LVEF), and left atrial diameter (LAD) (*P* > 0.05) (Figures 2(a)–2(c) and Table 2).

### 3.3. Effects of Liraglutide on the Induction Rate and Duration of AF

The CIH group showed a significantly higher induction rate and longer duration of AF compared to that in the control group substantially (50 ± 8.5% *vs*. 10 ± 6.8% and 7.99 ± 1.59 s *vs*. 0.53 ± 0.36 s, *P* < 0.05). After Lir administration, the induction rate and duration of AF reduced substantially (17 ± 8.0% *vs*. 50 ± 8.5% and 2.99 ± 1.64 s *vs*. 7.99 ± 1.59 s, *P* < 0.05) (Figures 3(a)–3(c)).

Among the parameters measured in the left atrium by epicardial electrical mapping, the left atrial (LA) conduction velocity decreased markedly while the absolute left atrial conduction heterogeneity increased in the CIH group compared to the control group (*P* < 0.05). After treatment with Lir, the left atrial conduction velocity increased (*P* < 0.05) but the absolute left atrial conduction heterogeneity showed no significant improvement (*P* > 0.05). Among the parameters measured in the right atrium, the right atrial conduction velocity reduced, while the absolute right atrial conduction heterogeneity increased in the CIH group (*P* < 0.05). Post-Lir administration, right atrial conduction velocity increased and the absolute right atrial conduction heterogeneity reduced significantly (*P* < 0.05) (Figures 3(d)–3(g)).

### 3.4. Liraglutide Ameliorates Atrial Fibrosis

HE staining showed a disorganized arrangement of atrial myocytes in the CIH group, which improved following Lir administration. Sirius red staining and Masson staining assays showed increased interstitial fibrosis in the atrial tissue in the CIH group compared to the control group and a significant reduction in interstitial fibrosis in the CIH+Lir group (Figures 4(a)–4(c)). The quantitative analysis of interstitial fibrous tissue in each group is shown in Figures 4(d) and 4(e). Fibrotic area in Masson among the control, Lir, CIH, and CIH+Lir groups was 2.46 ± 0.24%, 2.51 ± 0.25%, 12.37 ± 0.49%, and 6.41 ± 0.36%, respectively (*P* < 0.05). Fibrotic area in Sirius red among the control, Lir, CIH, and CIH+Lir groups was 1.98 ± 0.24%, 2.10 ± 0.29%, 9.53 ± 0.62%, and 5.57 ± 0.26%, respectively (*P* < 0.05). We also assessed the level of atrial fibrosis based on protein expressions. Compared to the CIH group, the protein level expressions of collagen III, collagen I, and ɑ-SMA were significantly higher in the CIH group (*P* < 0.05), while those of all fibrous proteins were significantly downregulated following Lir administration (*P* < 0.05), which was consistent with results pathological staining (Figures 4(f) and 4(g)).

### 3.5. Effects of Liraglutide on the Expression of miRNA-21 and Its Target Gene, PTEN

The expression of miRNA-21 was elevated in the CIH group compared to the control group, and the expression of PTEN, which was downstream target of miRNA-21, was attenuated in comparison with the control group, as demonstrated by the results of RT-qPCR (*P* < 0.05). However, Lir administration could reverse this trend significantly, with a decrease in miRNA-21 expression and an increase in the PTEN expression. Hence, Lir may regulate PTEN expression through its effect on miRNA-21 (Figures 5(a) and 5(b)).

### 3.6. Effect of Liraglutide on the PTEN/PI3K/AKT Signaling Pathway

To explore the potential mechanisms for the ameliorative effect of Lir on AR, we investigated the expression of the PTEN/PI3K/AKT signaling transduction pathway. In IHC experiments, positive reactions were mainly characterized by the presence of granules in the atrial tissues that are brownish-yellow, and the number and shade of these granules corresponded to the level of expression of the target protein. Relative to the control group, the expression of positive granules of PTEN decreased in the CIH group while those of PI3K and p-AKT increased significantly. Following the Lir administration, the expression of positive granules of PTEN increased and those of PI3K and p-AKT decreased substantially (*P* < 0.05); AKT expression was not statistically different among the groups (Figures 6(a) and 6(b) and Supplementary Table 2). We also observed changes in expression levels of proteins in the PTEN/PI3K/AKT signaling pathway by Western blotting. Compared to the control group, the PTEN expression level reduced significantly whereas those of PI3K and p-AKT were enhanced in CIH mice. Moreover, this trend was reversed by the administration of Lir (Figures 6(c)–6(f)).

### 3.7. Changes in Ion Channel and Gap Junction Proteins (CX43)

Compared to the control group, the protein expression of CACNA1C was found to be attenuated in the CIH group and Lir administration failed to ameliorate this effect. Moreover, the protein expression of KCNA5 did not show a statistically significant change among the four groups. In comparison to the control group, the expression of CX43 was markedly enhanced in the CIH group and could be reduced by Lir administration significantly (Figures 7(a)–7(d)).

### 3.8. Effects of Liraglutide on Inflammatory Marker Levels in Serum

Compared to the control group, the levels of both IL-6 and TNF-*α* were substantially elevated in the CIH group (34.08 ± 0.47 ng/L *vs*. 20.46 ± 0.85 ng/L and 51.22 ± 3.63 ng/L *vs*. 36.00 ± 1.38 ng/L, respectively, *P* < 0.05) and decreased significantly upon Lir administration (26.92 ± 1.25 ng/L *vs*. 34.08 ± 0.47 ng/L and 41.20 ± 2.16 ng/L *vs*. 51.22 ± 3.63 ng/L, respectively, *P* < 0.05) (Figures 8(a) and 8(b)).

## 4. Discussion

In this study, we aimed to assess whether Lir administration could ameliorate AAR, AER, and inflammatory responses induced by CIH. Herein, Lir was found to ameliorate the electrical conduction velocity and absolute heterogeneity of the atrium significantly and reduce the induction rate and duration of AF. In addition, Lir administration could reduce the area of fibrosis in the atria and attenuate the protein expressions of the fibrosis markers, collagen I, collagen III, and ɑ-SMA. Furthermore, the gene expressions of miRNA-21 and PTEN were regulated, and the downstream signaling pathway PI3K/AKT of PTEN was correspondingly altered following Lir administration. Lir reduced the levels of TNF-*α* and IL-6, the inflammatory factors in the serum, and reduced the expression of CX43. However, Lir administration did not ameliorate the reduction of CACNA1C protein expression induced by hypoxia. Overall, these results suggested that Lir could reduce CIH-induced AF by reducing the structural remodeling of the atria, i.e., by reducing atrial fibrosis and inflammatory responses.

Recent studies showed that OSA was closely associated with AF [22] and was a crucial risk factor for AF. In the treatment of AF, OSA can decrease the efficacy of catheter ablation, cardioversion, and antiarrhythmic drugs [12, 23]. CIH is a unique pathological mechanism of OSA, and the mechanism of CIH causing myocardial injury may be associated with an increase in metabolic abnormalities, sympathetic activity, oxidative stress, systemic inflammation, and endothelial dysfunction [11, 24]. Thus, in this study, we generated a mouse model of CIH and found that CIH could induce an increase in the mice's susceptibility to AF, along with a decrease in the atrial conduction velocity. Further pathological studies showed an increase in atrial fibrosis caused by CIH. Atrial fibrosis, as a crucial alteration in AR, is often used as an important component in the study of AF [25, 26]. In the present study, Lir ameliorated atrial fibrosis due to CIH by modulating the miRNA-21/PTEN/PI3K/AKT signaling pathway.

During the course of AF, miRNAs in the atrial tissue and blood flow had changed. A variety of miRNA molecules directly related to atrial fibrosis, such as miR-21, miR-101, and miR-208a/b. Cañón et al. demonstrated that elevated expression levels of miR-208a and miR-208b in the heart tissues of patients with atrial fibrillation [27]. miR-101 was shown to be protective and antifibrotic, and the mechanism of action includes inhibition of the expression of the proteins involved in the regulation of TGF-*β* signaling pathway [28]. Our previous study demonstrated that miR-21 is significantly upregulated in the CIH model [29]. Cardin et al. [30] demonstrate that knocking down miR-21 can inhibit the progression of atrial fibrosis and AF in rats. An *in vitro* study by Lorenzen et al. [31] demonstrated that angiotensin II stimulates AP-1 and promotes the transcriptional processes of miRNA-21, thereby targeting PTEN and Smad7 for degradation and leading to the activation of myocardial fibroblast and progression of myocardial fibrosis. Thus, miR-2l plays an important regulatory function in the development of myocardial fibrosis. PTEN is a downstream target of miR-21. It is a protease with phosphatidylinositol 3-phosphatase activity that antagonizes the action of P13K and has been found to possess a novel role as a fibrosis inhibitor. JMJD3 could preserve PTEN expression and thus protect against renal fibrosis by inhibiting the TGF-*β* and Notch signaling pathways [32]. Thus, the pathological processes of tissue fibrosis may be regulated by PTEN. PTEN is a recognized AKT inhibitor [33] and a potent negative regulator of the P13K/AKT signaling pathway. The PTEN/PI3K/AKT signaling pathway is implicated in several pathological and physiological activities, including apoptosis, cell proliferation, and cell differentiation. It is involved in the pathophysiological processes of several diseases [34]. Our results showed that Lir inhibited the high expression of miR-21 induced by CIH, increased the expression of PTEN gene and protein, and, thus, inhibited the phosphorylation of AKT. Hence, it was reasonable to conclude that Lir ameliorated atrial fibrosis, i.e., AAR by regulating miRNA-21/PTEN/PI3K/AKT signaling pathway.

Lir is a long-acting GLP-1 analog having 97% sequence homology with the human GLP-1. Increasing evidence suggested that Lir exerts cardiovascular effects in a direct or indirect manner. Lir reduces the risk factors for cardiovascular diseases by protecting the vascular endothelium from injury and inhibiting the apoptosis of cardiomyocytes, ameliorating cardiac ischemia-reperfusion injury, preventing atherosclerosis, improving blood pressure, lowering blood lipid levels, reducing body weight, and attenuating damage caused by chronic inflammatory responses [15, 19, 35]. Chen et al. [36] showed that Lir attenuates myocardial fibrosis in AngII-induced hypertensive mice by inhibiting ROS production. Sukumaran et al. [37] showed that Lir increases NO-mediated vasodilatation in the coronary microcirculation and ameliorates myocardial structural remodeling in an animal model of metabolic syndrome. These effects were not dependent on changes in body weight or blood glucose levels. It has been confirmed that Lir inhibited pressure overload-induced cardiac remodeling by modulating the PI3K/AKT and AMPK*α* signaling pathways, along with the suppression of the angiotensin-converting enzyme II [38]. A meta-analysis confirmed the beneficial effects of GLP-1-RA on major cardiovascular events, cardiovascular and all-cause mortality, stroke, and possibly myocardial infarction. In contrast, the effects on heart failure remain uncertain. Available data on atrial fibrillation seems to exclude any major safety issues in this respect [39]. In this study, we found that the protein expression levels of collagen III and collagen I, which are the markers of fibrosis, were attenuated significantly in CIH mice treated with Lir, which indicated that Lir could ameliorate atrial fibrosis.

AER refers to alterations in the expression and/or function of ion channel proteins on the membrane surface and gap junction proteins, as also the extracellular matrix structures. Electrophysiological changes underlie the induction of arrhythmias [40]. KCNA5 and CACNA1C are basic ion channels in the heart, generating ultrarapid delayed rectifier K^+^ current and inward L-type calcium current, respectively. These alterations in ion channels are crucial factors for the progression of AF [41]. CX43 is also associated closely with the progression and maintenance of AF [42]. Zhang et al. [43] reported that CIH causes a reduction in the expressions of CACNA1C and KCNA5. Ramadan et al. [44] showed that Lir ameliorated the abnormal expression of CX43 and reversed myocardial remodeling in diabetic rats. In this study, the protein expression of the CACNA1C was attenuated, while that of CX43 was elevated in the atrial tissues of CIH mice. Lir did not ameliorate the attenuated expression of CACNA1C but improved the abnormal expression of CX43 significantly. Thus, our study provided evidence of Lir-mediated amelioration of the abnormal CX43 expression induced by CIH.

The inflammatory responses play an important role in AF pathogenesis processes and alter AAR and AER. Lazzerini et al. [45] showed that systemic inflammation was a strong predictor of AF, which induced AER through elevated IL-6 levels and downregulated expression of cardiac connexins. Hogan et al. [46] reported that Lir can modulate the immune-mediated inflammatory response directly in diabetic patients by reducing the production of intercellular adhesion molecules and inflammatory cytokines, such as IL1, IL6, and TNF-*α*. In this study, the expressions of TNF-*α* and IL6, the inflammatory factors in the serum, were reduced significantly in CIH mice treated with Lir, which indicated that Lir could attenuate the inflammatory responses in CIH mice. Hence, we reasonably speculated that Lir ameliorated AR by attenuating the inflammatory responses.

In summary, our results suggested that hypoxia could lead to AR mainly with atrial fibrosis and increase the incidence rate of AF consequently. Lir could attenuate AR, and its mechanism of action may be linked to the regulation of the miRNA-21/PTEN/PI3K/AKT signaling pathway and suppression of the inflammatory responses.

## Figures and Tables

**Figure 1:** The effect of Lir on body weight, HW/BW, blood glucose, blood pressure, and heart rate. (a, b) Statistical results of the BW, HW/BW ratios (*n* = 8) after CIH and/or Lir treatment. BW was decreased following Lir administration. (c) The effect of Lir on blood glucose (*n* = 8), the blood glucose was decreased in the CIH+Lir group compared with the CIH group. (d–f) Heart rate and pressure measurements of systolic (SBP) and diastolic blood pressure (DBP) in different groups (*n* = 8). Both SBP and DBP were decreased with no change in HR following Lir administration. Data are mean ± SEM, ^∗^*P* < 0.05.

**Figure 2:** Echocardiography. (a) RV free wall thickness (RVFWT) measured by echocardiography from the parasternal short-axis view at the midpapillary level of the left ventricle. (b) Mean pulmonary artery pressure (mPAP), pulmonary acceleration time (PAT), and PAT/pulmonary ejection time (PET) ratios measured from pulmonary outflow PW Doppler tracings. (c) Representative parasternal long-axis views; M: mode views.

**Figure 3:** Lir reduces atrial fibrillation (AF) inducibility and AF duration induced by burst pacing and improves epicardial electrophysiological parameters. (a) Representative atrial electrogram recordings. Burst pacing is highlighted by solid underlines, whereas dashed underlines indicate AF. (b) Percentage of successful AF inducibility in each group (*n* = 6). (c) Average AF duration by burst pacing (*n* = 6). (d) Representative maps of spontaneous right atrial epicardial activation. (e) The comparison of right atrial (RA) epicardial conduction velocity, absolute inhomogeneity, and inhomogeneity index is detailed (*n* = 6). (f) Representative maps of spontaneous left atrial epicardial activation. (g) The comparison of left atrial (LA) epicardial conduction velocity, absolute inhomogeneity, and inhomogeneity index is detailed (*n* = 6). Data are mean ± SEM, ^∗^*P* < 0.05.

**Figure 4:** The effect of Lir on CIH-induced atrial fibrosis. (a–c) Representative images of HE, Masson, and Sirius red staining of atrial tissue in four groups. Interstitial fibrosis in the atrial tissue increased in the CIH group compared to the control group and reduced significantly in the CIH+Lir group. (d, e) Quantification of fibrotic area of Masson and Sirius red staining in four groups (*n* = 6). (f, g) Western blot analysis of the expression of collagen I, collagen III, and ɑ-SMA in the atrial. The expression of these proteins is increased in the CIH group compared to the control group and reduced in the CIH+Lir group (*n* = 6). Data are mean ± SEM, ^∗^*P* < 0.05.

**Figure 5:** mRNA expression levels determined by real-time fluorescent quantitative polymerase chain reaction for (a) miRNA-21 and (b) PTEN in four groups (*n* = 6). Data are mean ± SEM, ^∗^*P* < 0.05.

**Figure 6:** The effect of Lir on the PTEN/PI3K/AKT signaling pathways. (a) Representative photomicrographs of IHC-stained atrial sections from mice in four groups. The positive reaction primarily referred to the brown-yellow granules in the atrial tissues, the number and darkness of granules bespoken the expression levels of target proteins. (b) Mean option density (MOD) in four groups (*n* = 6). (c–f) Western blot analysis of the expression of PTEN, PI3K, and p-AKT/AKT in four groups (*n* = 6). Data are mean ± SEM, ^∗^*P* < 0.05.

**Figure 7:** The effect of Lir on the atrial electrical remodeling. (a–d) Western blot analysis of protein levels of CACNA1C, KCNA5, and CX43 (connexin 43) (*n* = 6). The increase in CX43 caused by CIH was ameliorated following Lir administration. Data are mean ± SEM, ^∗^*P* < 0.05.

**Figure 8:** The effect of Lir on inflammatory marker levels. (a, b) IL-6 and TNF-*α* in serum of mice detected by ELISA in four groups (*n* = 6). Both IL-6 and TNF-*α* increased after CIH and decreased significantly upon Lir administration. Data are mean ± SEM, ^∗^*P* < 0.05.

**Table 1:** Primers used for real-time PCR.

Gene	Primers (5′-3′)	Temperature (°C)
miRNA-21 stem-loop primer	GTCGTATCCAGTGCAGGGTCCGAGGTATTCGCACTGGATACGACATTTGG	75.04
miRNA-21 forward primer	GCCGAGCTGGTAAAATGGAA	56.00
Universal reverse primer	GTATCCAGTGCAGGGTCCGAGGT	63.77
U6	F: CTCGCTTCGGCAGCACA	56
	R: AACGCTTCACGAATTTGCGT	
GAPDH	F: GGCACAGTCAAGGCTGAGAATG	56
	R: ATGGTGGTGAAGACGCCAGTA	
PTEN	F: ACTGCAGAGTTGCACAGTATC	56
	R: GTCCGTCCTTTCCCAGCTTTA	

**Table 2:** Echocardiography parameters (*n* = 6).

	Control	Lir	CIH	CIH+Lir
RVFWT (mm)	0.33 ± 0.02	0.31 ± 0.03	0.46 ± 0.03^∗^	0.35 ± 0.02^#^
mPAP (mmHg)	67.27 ± 1.06	67.05 ± 1.10	72.13 ± 0.84^∗^	66.37 ± 0.92^#^
PAT (ms)	17.73 ± 0.60	17.47 ± 0.49	14.56 ± 0.53^∗^	16.81 ± 0.54^#^
PAT/PET	0.36 ± 0.02	0.36 ± 0.02	0.27 ± 0.02^∗^	0.34 ± 0.02^#^
LAD (mm)	1.99 ± 0.11	1.85 ± 0.10	2.01 ± 0.10	1.94 ± 0.11
LVEDD (mm)	4.37 ± 0.09	4.32 ± 0.13	4.29 ± 0.11	4.30 ± 0.20
LVEF (%)	57.79 ± 3.28	55.82 ± 2.77	54.46 ± 3.35	56.76 ± 2.96

Values are given as mean ± SEM. RVFWT: RV free wall thickness; mPAP: mean pulmonary artery pressure; PAT: pulmonary acceleration time; PAT/PET: PAT/pulmonary ejection time (PET) ratios; LAD: left atria diameter; LVEDD: left ventricular end-diastolic dimension; LVEF: left ventricular ejection fraction. ^∗^Significant difference between the control and CIH groups at *P* < 0.05. ^#^Significant difference between CIH and CIH+Lir groups at *P* < 0.05.

## Data Availability

The original contributions presented in the study are included in the article. Further inquiries can be directed to the corresponding authors.

## Supplementary Materials

Supplementary Materials Supplementary Table 1: baseline and hematological parameters. Supplementary Table 2: mean option density (MOD) in four groups.
